The article "Progressive Rain Removal Based on the Combination Network of CNN and Transformer" was published in 2022. Journal: Comput Intell Neurosci.

# Progressive Rain Removal Based on the Combination Network of CNN and Transformer

**DOI:** 10.1155/2022/5067175

**Published:** 2022-09-24

**Authors:** Tianming Wang, Kaige Wang, Qing Li

**Affiliations:** ^1^Intelligent Manufacturing Electronics Research Center, Institute of Microelectronics of the Chinese Academy of Sciences, Beijing 100083, China; ^2^School of Integrated Circuits, University of Chinese Academy of Sciences, Beijing 100083, China

## Abstract

The rain removal method based on CNN develops rapidly. However, convolution operation has the disadvantages of limited receptive field and inadaptability to the input content. Recently, another neural network structure Transformer has shown excellent performance in natural language processing and advanced visual tasks by modeling global relationships, but Transformer has limitations in capturing local dependencies. To address the above limitations, we propose the combination network of CNN and Transformer, which fully combines the advantages of CNN and Transformer structure to complete the task of image restoration. We use CNN to provide preliminary output and adopt Transformer architecture to further optimize the output of CNN. In addition, by using some key designs in module connection, our model strengthens feature propagation and encourages feature reuse, allowing better information and gradient flow. The experimental results show that compared with the existing methods, our method can remove the rain lines more comprehensively and achieve the state-of-the-art results. Besides, the experimental results also demonstrate that the CNN structure can be effectively combined with Transformer to fully utilize the superiority of different structures.

## 1. Introduction

In recent years, advanced computer vision tasks such as image classification [1], object detection [2], and object tracking [3] have made great progress, and are widely used in real life, such as intelligent monitoring, driverless, and so on. However, the performance of these models will be seriously affected in the case of bad weather such as rain, snow, and fog. It is very important to seek solutions to acquire high-quality images in bad weather conditions. In this paper, we solve the problem of removing rain from a single image. The imaging model of rainy days can be simply formulated as a linear combination of rainless image *B* and rain steak image *R*.

(1) $$\begin{array}{c} O=B+R\text{,} \end{array}$$

where *O* represents the raw data obtained by the camera. The rain removal task refers to separating the rain-free image *B* from *O* as shown in Figure 1. This is an ill-posed problem, because the same *O* can be generated by different *B* and *R* pairs. Therefore, how to get high-quality rain removal image is an important problem to be solved in computer vision tasks.

Image rain removal is a very hot topic. Some methods [4–6] focus on removing the rain steaks in the video. Such methods make full use of the sequence relationship of continuous frames in video data. However, for single image rain removal, there is no continuous time series and can only use spatial context information, so it is more challenging. Single image rain removal went through an evolutionary process of moving from model-driven to data-driven. Model-driven methods are subdivided into filter-based methods and prior knowledge-based methods. In the filter-based methods represented by [7, 8], researchers have preliminary achieved image rain removal by analyzing the frequency characteristics of rain lines and backgrounds, and designing filters with specific structures or weights to obtain rain removal images. Based on prior knowledge, the rain removal method utilizes available mathematical methods and analytical techniques, such as morphological component analysis [9], sparse coding [10], dictionary learning [11], and GMM prior knowledge [12] to distinguish the raindrops from the background. However, the above methods have common drawbacks, including high computational complexity, long running time, and incomplete rain removal results.

With the proposal and rapid development of convolutional neural networks, data-driven methods have shown amazing results in various computer vision fields, and single-image rain removal using deep learning techniques has received widespread attention. These methods focus on designing various depth neural networks. Inspired by ResNet, a depth detail network [13] is proposed to remove high-frequency rainfall content, as well as a large-scale synthetic data set composed of rain/rainless image pairs. Some multilevel [14, 15] or multistream [16] network structures have been proposed to learn multiscale rain layer information. Due to the powerful learning ability of generative adversarial networks (GAN), some methods based on GAN structure [17, 18] have been proposed to realize the task of rain removal. Recently, some scholars proposed a series of new methods [19–21], which greatly improved the model performance. A recurrent strategy [19] is proposed to complete the rain removal task in which a recursive layer is introduced to take advantage of the dependence of the deep features of different stages. Aiming at the optimization process of the model, a model-driven deep neural network [20] has a completely interpretable network structure. MPRNet [21] proposed a multistage architecture, which gradually learns the recovery function to decompose the whole recovery process into more manageable steps. These methods take CNN network as the backbone and convolution as the basic operation. With its local connectivity and translation invariance, convolution is very suitable as a feature extractor of image data. However, there are still some problems in convolution operation. First, the convolution operator has a limited receptive field. The pixel in the image can only capture the information of its surrounding pixels and cannot model the dependence of long-distance pixels. Second, convolution operation has static weight, so the interaction between image and convolution kernel is independent of image content. Using the same convolution kernel to restore different image regions may not be the best choice. Due to the limitation of convolution operation, CNN architecture cannot achieve the ideal effect of rain removal.

To break through the limitation of convolution, an ideal method is to adopt self-attention (SA) mechanism, which is the core component of Transformer [22]. Transformer performs well in natural language processing. Since Vit [23] introduced it into vision tasks, its potential is being tapped. SA models the relationship between pixels by calculating the correlation matrix with all other positions, so it can obtain the global receptive field. In addition, the calculation of attention map is a dynamic mechanism, because the correlation matrix will depend on the input. Based on this, Transformer has the advantages that CNN does not have. However, local context information is also very important for image restoration tasks, because the neighborhoods of degraded pixels can be used to restore its clean version, but some work shows that Transformer has limitations in capturing local dependencies.

For the rain removal task, the model requires both global information to know where the rain line is and detail information to restore it. However, a single CNN or Transformer structure does not have both properties. If both structures are included in the model, it can capture local dependencies to improve the inference of content and capture global information to improve the inference of location. In this paper, inspired by the progressive step [21], we propose a combination network of CNN and Transformer (CNCT). Specifically, our rain removal network includes two subnetworks: Net-C and Net-T. Net-C, as the first stage of the network, takes CNN as the backbone architecture. This network adopts single-scale channel to provide spatially accurate output. Net-T is the second stage of the network, with Transformer structure as the backbone architecture. It takes the depth feature of the first-stage output as the input and uses the attention mechanism to capture the global interaction of the context and further optimize the semantic details. We show that the combination of these two design options is effective for image restoration in a multistage architecture.

In addition, we prove that simply transferring the final output from the first stage to the second stage cannot get the best effect. Thus, our basic unit in Net-T not only has SA module but also includes cross-attention (CA) module, which is a cross-stage attention mechanism by spreading semantic features from early to late. In addition, this method simplifies the information flow between stages and effectively stabilizes the multistage network optimization.

For this paper, the main contributions are as follows:

1. CNN is good at capturing local dependencies but has a limited receptive field, while Transformer is the opposite. For the rain removal task, the model requires both global information to know where the rain line is and detail information to restore it. Thus, we propose a new multistage method combining CNN and Transformer, which can generate rich context and accurate spatial output.
2. To strengthen feature propagation, encourage feature reuse, and avoid losing information, we propose a cross-stage attention mechanism, which aggregates the features of different stages.
3. We demonstrated the effectiveness of our CNCT on multiple synthetic and real-world datasets, and we also provided detailed ablation and qualitative results.

## 2. Related Work

In this section, we briefly review the network structure used in the proposed network. Specifically, we introduce the applications of CNN and Transformer in recent years.

### 2.1. CNN Structure

In the past decade, neural networks, especially CNN, have made great progress and influence [24]. Although the method of back-propagation-trained network has been proposed in the 1980s, neural networks did not become the focus until AlexNet [25] won the champion of ImageNet competition in 2012. Since then, CNN has made great achievements in the field of image processing and computer vision, and some representative networks have been proposed, such as VGGNet [26], Inceptions [27], ResNe(X)t [28, 29], DenseNet [30], MobileNet [31], and EfficientNet [32]. They focus on different aspects of accuracy, efficiency, and scalability, and promote many useful design principles. It is not accidental that CNN is suitable for image processing. The shared convolution kernel parameters and the sparsity of interlayer connections enable CNN to learn grid topology features with less computation and stable effect. Specifically, convolution has a salient ability to extract features from image and has the characteristics of translation invariance. It can recognize similar features in different positions in space. When used in sliding window mode, computing is shared, so CNN is also efficient. Because of this characteristic, CNN is widely used in computer vision applications, such as image classification [1], object detection [2, 33, 34], object tracking [35], semantic segmentation [36], image painting [37], image restoration [21, 38], and image generation [39].

### 2.2. Vision Transformers

Transformer [22] has remarkable performance in natural language processing. Different from CNN's local perception, the Transformer-based network captures the long-term dependence on the input data by calculating the global attention matrix, which also inspired computer vision researchers. Vit [23] uses a pure Transformer structure and achieves better results in image classification than the state-of-the-art CNN through large-scale data pretraining. After that, Transformer was also applied to advanced computer vision tasks such as object detection [40] and image segmentation [41]. The remarkable characteristic of these models is that they have a strong ability to learn the long-term dependence between image patch sequences, and are adaptive to the given input content. Although there are many explorations in the field of vision, the introduction of Transformer into low-level vision still lacks of exploration because of its complexity growing quadratically with the spatial resolution. One potential approach is to use Swin Transformer [42], which limits the calculation of attention matrix to local windows. These methods for image restoration cannot obtain the global receptive field, which is contrary to the original intention of using Transformer. Restormer [43] proposes a Transformer model that can learn long-term dependencies while maintaining computational efficiency. The Transformer model we used in this paper will follow the Restormer paradigm, which proves to be effective for image restoration.

## 3. Methods

In this section, we propose a progressive rain removal network as shown in Figure 2. The whole network process procedure is shown in Algorithm 1. The network consists of two subnetworks: Net-C and Net-T. Net-C takes CNN as the backbone, and Net-T takes Transformer as the backbone. Each unit of Net-T receives the output of the corresponding unit of Net-C as well as the previous unit as input. Next, we will introduce the components of the proposed method in detail.

### 3.1. Net-C

The architecture of Net-C is shown in the upper half of Figure 2. We will introduce the process of Net-C in detail.

First, for the input image ∈*R*^*H*×*W*×3^, it will be processed by a convolution operation in which both convolution kernel and stride are *p* and the number of channels is *C*_*di* *m*_. In this process, the *p* × *p* pixels in the image form a noncoincident patch and will be mapped from the image space to original feature maps *F*_0_ ∈ *R*^*H*/*P*×*W*/*P*×*C*_di m_^, which is defined as follows:

(2) $$\begin{array}{c} F_{0}={Conv}_{p\times p}\left(O\right)\text{.} \end{array}$$

Dividing the image into patches will not change the original image itself, but divides the original large image into small images. The resolution of the image becomes 1/*P* of the original. This operation greatly improves the processing efficiency. In our implementation, we use *p* = 2 and *C*_di m_ = 48.

Then, *F*_0_ will be sent into the basic unit sequence of Net-C, which adopts the mode of dense connection. Dense connection is an efficient architecture because it can enhance the transmission of feature streams. Net-C unit is composed of a series of dense blocks (DB), which is as shown in Figure 3. For the *l*-th DB, it concatenates the aggregated feature maps of the past *l* − 1 DBs and compresses them into *C*_di m_ dimension:

(3) $$\begin{array}{c} f_{l}={conv}_{1\times 1}\left(Concat\left[X_{0},X_{1},\cdots X_{l-1}\right]\right)\text{,} \end{array}$$

where Concat[*X*_0_, *X*_1_, ⋯*X*_*l*−1_] refers to the concatenation of the aggregated feature maps produced by *DB*_0_, *DB*_1_, ⋯*DB*_*l*−1_. We directly use a 1 × 1 convolution to compress the channel. The compression operation greatly reduces the parameters of DB. Then, the compressed feature maps will be further aggregated and compressed with the output of the previous DB to obtain the aggregated feature maps *X*_*l*_ ∈ *R*^*H*/*P*×*W*/*P*×*C*_di m_^ of the current DB:

(4) $$\begin{array}{c} X_{l}={conv}_{1\times 1}\left(Concat\left[F_{l-1},f_{l}\right]\right)\text{.} \end{array}$$

This process also uses 1 × 1 convolution to reduce parameters. The obtained aggregated features will be further processed by a residual network. Finally, the output of the current DB will be obtained.

(5) $$\begin{array}{c} F_{l}={conv}_{3\times 3}\left(GELU\left({conv}_{3\times 3}\left(X_{l}\right)\right)\right)+X_{l}\text{.} \end{array}$$

The residual network includes two 3 × 3 convolution layers and the GELU activation function, in which the first convolution layer increases the number of channels by 4 times and the second convolution layer restores the number of channels. We stack *n* DBs to get Net-C unit. *K* Net-C units are stacked to obtain the backbone of Net-C. *F*_0_ is transformed into the final depth feature *F*_*k*_ after Net-C unit transmission and processing one after another. In our implementation, we use *K* = 5 and the corresponding *n* is (3, 3, 3, 3, 4).

Finally, in our restoration part, we first use a set of convolution layers to convert the number of depth feature channels to 3*p*^2^ and then use Pixel shuffle operation and residual structure to transform it into rainless image *B* ∈ *R*^*H*×*W*×3^ as

(6) $$\begin{array}{c} B=Pixelshuffle\left(convs\left(F_{k}\right)\right)+O\text{ .} \end{array}$$

In our implementation, convs consists of two convolution layers, of which the first maintains the number of channels and the second performs channel conversion.

### 3.2. Net-T

The architecture of Net-T is shown in the lower half of Figure 2. It is composed of a series of Net-T units as shown in Figure 4. We use two attention patterns: self-attention and cross-attention. After the attention calculation is completed, we use a feed-forward network (FFN) for further feature transformation. This module uses two 3 × 3 convolution layers with GELU activation function between them. We add a LayerNorm (LN) layer after SA, CA, and FFN, and all modules use a residual connection. The whole unit has three steps as follows:

(7) $$\begin{array}{c} X=SA\left(\text{LN}\left(X\right)\right)+X\text{,}\\ X=CA\left(\text{LN}\left(X\right),Y\right)+X\text{,}\\ X=FFN\left(\text{LN}\left(X\right)\right)+X\text{,} \end{array}$$

where *Y* is the output of feature maps from the first stage of the corresponding unit.

Next, we will introduce the attention component of the Net-T unit in detail.

#### 3.2.1. Self-Attention Module

It is very difficult to apply Transformer directly to image restoration. The standard Transformer will calculate the correlation matrix between all locations. For input feature map ∈*R*^*H*×*W*×*C*^, we can get *Q*, *K* ∈ *R*^*HW*×*C*^ in standard Transformer. The multiplication calculation times of calculating the attention map have quadratic complexity with the image resolution as

(8) $$\begin{array}{c} \Omega \left(QK^{T}\right)={\left(HW\right)}^{2}C\text{.} \end{array}$$

It is not appropriate to use a standard Transformer on a high-resolution feature map. Swin Transformer calculates attention map on the local window and continuously expands the receptive field by moving the window. However, this is not in line with our intention to adopt the global receptive field. Following Restormer [43], we introduced transposed attention to replace vanilla SA.

The SA module based on transposed attention is shown in Figure 5(a), and its pseudocode based on PyTorch is shown in Algorithm 2. In our implementation, for a given input ∈*R*^*H*×*W*×*C*^, SA will first generate *Q*, *K*, *V* ∈ *R*^*HW*×*C*^ by 3 groups of 1 × 1 convolution and 3 × 3 depthwise convolution and reshape operation yielding:

(9) $$\begin{array}{c} Q=R\left({Dconv}_{3\times 3}\left({conv}_{1\times 1}\left(X\right)\right)\right)\text{,}\\ K=R\left({Dconv}_{3\times 3}\left({conv}_{1\times 1}\left(X\right)\right)\right)\text{,}\\ V=R\left({Dconv}_{3\times 3}\left({conv}_{1\times 1}\left(X\right)\right)\right)\text{,} \end{array}$$

where *R* represents reshape operation. Unlike vanilla SA, we calculate the attention map on the feature channel rather than in the spatial dimension. Specifically, instead of calculating *QK*^*T*^, we calculate *K*^*T*^*Q* to obtain attention map ∈*R*^*C*×*C*^, rather than the standard attention map ∈*R*^*HW*×*HW*^. This method has the following advantages: first, the number of multiplication calculations required to calculate *K*^*T*^*Q* has linear complexity with image resolution as

(10) $$\begin{array}{c} \Omega \left(K^{T}Q\right)=HWC^{2}\text{.} \end{array}$$

In addition, it implicitly models the global relationship between pixels.

Thus, the process of SA is defined as

(11) $$\begin{array}{c} \hat{X}=V\cdot Softmax\left(\frac{K^{T}Q}{d}\right)\text{,} \end{array}$$

where $\hat{X}$ is the output of SA module and *d* is a parameter that can be learned. We use a multihead attention mechanism following Restormer, and we set the number of heads as 2.

#### 3.2.2. Cross-Attention Module

CA module is another attention component of the Net-T unit. Unlike SA, CA has two parts of the input. One part is the output feature *X* of the previous step, and the other part is the output feature *Y* from the corresponding unit of the first stage as shown in Figure 2. To correspond to the first stage, Net-T and Net-C have the same number of units.

The function of the CA module is to interact the semantic features of Net-T and Net-C. The processing flow is similar to the SA module. Except that the acquisition methods of *Q*, *K*, and *V* are different, the other procedures will be exactly the same. In CA module, *Q* comes from *X*, while *K* and *V* come from *Y* as

(12) $$\begin{array}{c} Q=R\left({Dconv}_{3\times 3}\left({conv}_{1\times 1}\left(X\right)\right)\right)\text{,}\\ K=R\left({Dconv}_{3\times 3}\left({conv}_{1\times 1}\left(Y\right)\right)\right)\text{,}\\ V=R\left({Dconv}_{3\times 3}\left({conv}_{1\times 1}\left(Y\right)\right)\right)\text{.} \end{array}$$

Figure 5(b) shows the idea of our cross-attention, where the fusion involves the *X* and *Y*. Its pseudocode based on PyTorch is shown in Algorithm 3. In particular, because *X* has learned its own abstract information in the SA step, interacting with *Y* helps to get information at a different stage. Based on the characteristics of Transformer, the CA module can selectively receive the results of the first stage, provide supplementary information for the current output results, and avoid redundant information. CA has several advantages. First, it helps to spread contextual features from Net-C to Net-T. Second, the features of one stage help to enrich the features of the next stage. Third, the network optimization process becomes more stable because it simplifies the flow of information.

### 3.3. Loss Function

For the input rain image *O*, our network will finally output the corresponding rain removal image $\hat{B}$, We use negative SSIM loss to optimize this process. SSIM measures the similarity of two images according to their brightness, contrast, and structure. The larger the SSIM value, the better the image restoration quality. However, to better train the network and make it converge, the negative value of SSIM needs to be considered in loss calculation as

(13) $$\begin{array}{c} L_{SSIM}=-SSIM\left(\hat{B},B\right)\text{,} \end{array}$$

where *B* is ground truth. Specifically, both stages will output the rain removal image $\hat{B_{i}\;,}i=1,2\text{.}$ We apply SSIM loss to the rain removal image at each stage. In addition, to improve the rain removal effect of the model, during the training process, the output feature maps of each unit are restored to the rain removal image $\hat{B_{ij}\;}\left(i\right.=1,2,j=1,2,\cdots k\text{,}$ where *k* is the number of units in the network through the restoration module. We impose additional SSIM loss on it. The loss of the whole network can be written as

(14) $$\begin{array}{c} L_{SSIM}=\overset{k}{\underset{j}{\sum }}a_{1}\;SSIM\left(\hat{B_{1j}\;},B\right)+a_{2}SSIM\left(\hat{B_{1k}\;},B\right)+\\ \;\overset{k}{\underset{j}{\sum }}b_{1}\;SSIM\left(\hat{B_{2j}\;},B\right)+b_{2}SSIM\left(\hat{B_{2k}\;},B\right)\text{.} \end{array}$$

To ensure the quality of the final rain removal image, we add additional loss to the output of the last unit of each stage. The whole loss function consists of four hyperparameters *a*_1_, *a*_2_, *b*_1_, *b*_2_. In our implementation, *a*_1_=0.1, *a*_2_=1, *b*_1_=0.1, *b*_2_=1.

## 4. Experiments

In this section, we conduct ablation experiments on the structure of the proposed CNCT and compare it with the state-of-the-art methods to verify the effectiveness of the proposed method. Our ablation experiments include the verification of CA and SA modules, the impact of loss function, and the necessity of the combination of the two networks. Then, we compare our network with the results of some state-of-the-arts.

Our network is implemented in PyTorch. Training and testing were carried out on an NVIDIA Tesla V100 32G. Our network follows the settings of the previous work [19, 44]. Specially, we use a sliding window with a size of 112 and a sliding step of 96 to segment the image into patches. During training, batch_size is 16 and the initial learning rate is 1e − 3. The whole network trains 100 epochs, and when reaches at 30, 50, and 80 epoch, the learning rate decreases by 5 times. All tests were performed using the final epoch results.

### 4.1. Ablation Experiment

All ablation experiments were performed on Rain100H [14]. The training set includes 1800 images, and the test set includes 100 images. We use the average PSNR and SSIM of 100 test images as the evaluation results.

Attention module: the Transformer structure we use includes two parts: SA and CA. To verify the importance of these two parts, we performed ablation experiments on the role of each part.  Table 1 shows the average PSNR and SSIM results of rain removal images of different transformer structures obtained on Rain100H. First, we retained SA and removed CA, resulting in a decrease of PSNR by 0.27 dB. When CA was retained and SA was removed, PSNR decreased by 0.30 dB. This shows that SA and CA are both necessary for our Transformer structure. They work together to make it have a stronger image restoration ability.

Loss function: in the deep learning task, the design of loss function will have a great impact on the final result.  Table 2 compares the average PSNR and average SSIM values obtained on Rain100 H after 100 epoch training with different hyperparameters *a*_1_, *a*_2_, *b*_1_, and *b*_2_. It can be seen from rows 1 and 5 that it is necessary to apply loss to the first stage; otherwise, Transformer cannot optimize the output. In the second row, we set *b*_1_ and *b*_2_ to 0; that is, we only trained Net-C but not Net-T. We use the output of Net-C as the final output. It can be seen that the PSNR trained with CNN and transformer is 0.64 dB higher than that trained with CNN only. In the third row, we set *a*_1_ and *b*_1_ to 0 and PSNR decreased by 0.91 dB, indicating that adding additional loss after each unit can produce a better rain removal effect.

Transformer vs. convolution: to verify the necessity of combining CNN with Transformer, we replaced all the attention modules in Net-T with 3 × 3 convolution, while keeping the others unchanged. The experimental results are shown in Table 3. It can be seen that using Transformer is 0.80 dB higher than using CNN. This research indicates that the reason for performance improvement is not by increasing the network depth. Compared with the original convolution block, the proposed combination metric is effective.

### 4.2. Evaluation on Synthetic Datasets

It is impractical to obtain the images of rainy days and the corresponding images of no rain in the real scene. Therefore, we train and test CNCT on synthetic image pairs. We train models on RainTrainH [14] and RainTrainL [14], corresponding to RainTrainH and RainTrainL training models of heavy rain and light rain images, respectively. The RainTrainH training model was tested on Rain100H, Rain200H, and Rain12 [45], and the RainTrainL training model was tested on Rain100L.

In order to prove the superiority of CNCT, we compare our method with the traditional method GMM [12] and the state-of-the-art deep learning methods RESCAN [46], PreNet [19], RMUN [47], TS-CGAN [48], LSPN [49], SSDRNet [50], MPRNet [21], and Restormer [43]. MPRnet is a multistage CNN architecture, and Restormer is a pure Transformer architecture. For GMM, we directly run the open source code and obtain the test results of the above test set.

Since the code of methods [47–49] cannot be obtained, we refer to some comparison results given in their paper. For other methods, if there is no pretrained model, we use the implementation provided by the author to retrain it. For Restormer, we use an unofficial reproduction version (https://github.com/leftthomas/Restormer). Following [21], we calculate SSIM and PSNR in YCbCr channel.

Table 4 shows the average PSNR and average SSIM values of the results obtained by our method and other methods on different data sets. In Table 4, the data marked with black and underlined represent the first and second levels, respectively. It can be seen from the table that our CNCT has the highest average PSNR and SSIM values on Rain100H and Rain100 L. On Rain200H and Rain12, we achieved comparable results. It is worth pointing out that CNCT has only 4.0 M parameters, whereas Restormer has 26.1 M, which is a so large model. This shows that our structure is very efficient in learning feature representation for image recovery.

Figure 6 shows the rain removal results on two groups of Rain100H test sets. We only show the methods that can be reproduced or have been open source. It can be seen the result of CNCT is obviously superior to other methods in visual effect and detail maintenance. The traditional algorithm GMM has some shortcomings in the ability of removing rainstorms. Neural network-based methods RESCAN, PreNet, and SSDRNet improved the performance but were limited. As state-of-the-art methods, MPRNet and Restormer still have some defects in maintaining details. In the enlarged area, we can see that there are some blurs in the restoration image. For example, the texture details in the restoration of letters and fences are not very satisfactory. Our method not only removes the rain lines but also retains the edge information, which is basically consistent with the real value of the ground.

### 4.3. Evaluation on Real-World Datasets

In the previous section, we showed that our model achieves the best performance on synthetic datasets. However, in natural scenes, rain lines are more complex. Following [14], we test the effectiveness of removing rain lines in natural scenes on the model trained on RaintrainH.

Figure 7 shows the rain removal effect of our model on real-world datasets. Since there is no ground truth corresponding to the real scene, we only compare our model with other models in terms of subjective visual effects. It can be seen that the rain removal effect of other methods is not ideal, and there are many residual traces. In addition, there are fuzzy and low-quality visual effects in the removal results. Our method removes rain lines as much as possible while retaining more details.

## 5. Conclusions

This paper proposes an end-to-end rain removal network by combining CNN and Transformer structure. This network consists of two subnetworks: Net-C and Net-T, which are used for single rain removal. We fully combine the advantages of CNN and Transformer to achieve a better rainwater removal effect. Net-C adopts CNN architecture, providing spatially accurate but semantically unreliable output. Net-T adopts Transformer architecture to further optimize the output of the previous subnetwork. We use cross-attention combined with skip connection to achieve better information flow transmission so that the network can make full use of shallow information to complete the rain removal task. A large number of experimental results show that our method has a better effect than the state-of-the-art methods. Besides, the experimental results also demonstrate that the CNN structure can be effectively combined with Transformer to fully utilize the superiority of different structures. This provides a new approach to building diverse networks for many researchers who are limited by the drawbacks of CNN or Transformer. In future research, it is also important to explore the application of this network in other image restoration tasks.

## Figures and Tables

**Figure 1:** An example of rain removal.

**Figure 2:** The architecture of CNCT. The input image will go through two stages: Net-C and Net-T. Net-C is a convolutional neural network, which first maps the image into depth features by shallow feature extraction module, and then continues processing by a succession of Net-C units. Net-T adopts the Transformer structure, which takes the output of the last Net-C unit as the input and processes it by a succession of Net-T units. There is a cross-stage feature fusion mechanism (pink arrows) between the corresponding units in different stages. Finally, image reconstruction module restores the depth features to images.

**Figure 3:** The architecture of dense block. There are two 1 × 1 convolution layers in this module. The first convolution realizes the aggregation of past features, and the second convolution aggregates the aggregated past features and current features. Then, the features will be processed by a residual network.

**Figure 4:** The architecture of Net-T unit. We use two attention patterns: self-attention and cross-attention. After the attention calculation is completed, we use feed-forward network (FFN) for further feature transformation.

**Figure 5:** The architecture of self-attention module and cross-attention module. *R* means reshape operation; *S* means softmax operation; × means matrix multiplication. “Left” means to the left of the operator, while “right” means to the right of the operator. (a) The architecture of self-attention module and (b) the architecture of cross-attention module.

**Figure 6:** Image deraining results on synthetic datasets.

**Figure 7:** Image deraining results on real-world datasets.

**Algorithm 1:** Model process procedure.

**Algorithm 2:** SA process procedure.

**Algorithm 3:** CA process procedure.

**Table 1:** The influence of attention module.

SA	CA	PSNR	SSIM
√		32.17	0.940
	√	32.14	0.939
√	√	32.44	0.942

**Table 2:** The results of different hyperparameters in loss function.

a1	a2	b1	b2	PSNR	SSIM
0	0	0.1	1	29.84	0.908
0.1	1	0	0	31.80	0.934
0	1	0	1	31.53	0.933
0	0	0	1	29.40	0.907
0.1	1	0.1	1	32.44	0.942

**Table 3:** Comparison of different network architectures.

Module	PSNR	SSIM
CNN	31.64	0.931
Transformer	32.44	0.942

**Table 4:** Image deraining results.

Models	Rain100H	Rain200H	Rain12	Rain100L	Average
GMM	15.05/0.425	14.71/0.438	32.02/0.855	28.66/0.865	22.61/0.646
RESCAN	26.94/0.850	26.11/0.844	33.27/0.953	33.97/0.955	30.07/0.901
PreNet	29.47/0.903	28.74/0.899	36.50/0.970	37.04/0.978	32.94/0.938
SSDRNet	30.87 0.913	30.25/0.911	35.96/0.944	39.15/0.984	34.05/0.938
TS-CGAN	26.87 0.849	—	—	36.61/0.975	—
LSPN	26.87/0.850	—	—	37.18/0.980	—
MPRNet	31.49/0.925	29.98/0.917	37.47/0.973	38.28/0.981	34.31/0.949
RMUN	28.99/0.905	—	—	38.21/0.984	—
Restormer	31.96/0.916	**30.75**/0.911	37.92/**0.975**	39.98/0.987	35.15/0.947
CNCT (ours)	**32.44**/**0.942**	30.26/**0.923**	**37.92**/0.974	**40.58**/**0.989**	**35.30**/**0.957**

Best and second-best scores are highlighted and underlined.

## Data Availability

The data used to support the findings of this study are included within the article.
